# Design and Practical Application of Sports Visualization Platform Based on Tracking Algorithm

**DOI:** 10.1155/2022/4744939

**Published:** 2022-08-16

**Authors:** Xia Hua, Lei Han

**Affiliations:** Department of Physical Education, China University of Petroleum (East China), Qingdao, Shandong 266580, China

## Abstract

Machine learning methods use computers to imitate human learning activities to discover new knowledge and enhance learning effects through continuous improvement. The main process is to further classify or predict unknown data by learning from existing experience and creating a learning machine. In order to improve the real-time performance and accuracy of the distributed EM algorithm for machine online learning, a clustering analysis algorithm based on distance measurement is proposed in combination with related theories. Among them, the greedy EM algorithm is a practical and important algorithm. However, the existing methods cannot simultaneously load a large amount of social information into the memory at a time. Therefore, we created a Hadoop cluster to cluster the Gaussian mixture model and check the accuracy of the algorithm, then compare the running time of the distributed EM algorithm and the greedy algorithm to verify the efficiency of the algorithm, and finally check the scalability of the algorithm by increasing the number of nodes. Based on this fact, this article has conducted research and discussion on the visualization of sports movements, and the teaching of visualization of sports movements can stimulate students' interest in physical education. The traditional physical education curriculum is completely based on the teacher's oral explanation and personal demonstration, and the emergence of visualized teaching of motor movements broke the teacher-centered teaching model and made teaching methods more interesting. This stimulated students' interest in sports and improved classroom efficiency.

## 1. Introduction

In recent years, many researchers at home and abroad have been studying machine learning algorithms, and due to the diversity of target information observed in the machine learning process, machine learning is still a difficult problem [1]. Recently, the application of machine learning theory in distributed EM algorithms has become a research hotspot [2]. Different from traditional learning, the purpose of machine learning for the EM algorithm is to convert the greedy EM algorithm for distributed processing (i.e., use the target algorithm for background classification of the target), process each node, and generate the corresponding key-value pair. One of the main characteristics of machine learning is learning, even though computers have the same “learning” capabilities as humans [3]. It can repair the state of the machine in time by identifying various changes in the EM algorithm, and these changes are applicable to different problems in the EM algorithm. Specifically, the mapper performs data distribution, processes each node, and generates corresponding key-value pairs, and then superimposes the generated key-value pairs [4]. Finally, the optimal Gaussian mixture model that satisfies the convergence condition is obtained. Then, the number of components in the Gaussian mixture model is obtained accordingly. Finally, the three sets of experimental results show that the algorithm significantly improves the speed of calculation, can meet the processing of multiple data sets, and have great advantages under the condition of ensuring that the number of model components is not required in advance and the number of model components can be accurately obtained [5]. And it has good robustness and algorithm scalability. On this basis, this article analyzes and studies the visualization of sports movements. Movement visualization teaching method can effectively reduce the time for teachers to demonstrate and explain actions, so that teachers can spend more of their free time on teaching itself, thereby helping teachers find and solve students' problems in time, and guide students to learn effectively [6, 7]. Teachers can pay more attention to students, which will also help improve teachers' reflection after the course and provide materials for academic research [8]. Movement visualization teaching resources themselves are also good academic research materials. Teachers can use the teaching experience of studying visual teaching to improve their own teaching level. In addition, visual teaching can enrich teaching resources and be provided to teachers as a new teaching idea [9]. It can be seen that the application of action visualization teaching in sports courses is of great significance. Movement visualization teaching resources are the core of teachers' movement visualization teaching, so this research is very necessary.

## 2. Related Work

The literature introduces the MapReduce rendering framework model and the big data platform distributed by Hadoop [10]. It includes the working principle of the MapReduce framework, working model and program model, as well as a detailed study of the HDFS architecture and file reading and writing process [11]. The literature introduces the Hadoop cluster and confirms the accuracy of the Gaussian mixture grouping model. According to the algorithm in this paper, comparing the time-consuming of the traditional EM algorithm and the greedy algorithm, the effectiveness of the algorithm is verified. Finally, the scalability of the algorithm is verified by increasing the number of nodes [12]. The literature introduces the basic principles of the Haar-like form used in the algorithm and analyzes several classical algorithms for tracking research targets. In order to solve the problem that the selected weak classifiers cannot be distinguished from the target samples, it proposes to weight the weak classifiers according to the selection order [13]. For positive samples, according to the selected strategy, more weights are assigned to samples that are more similar to the target, and the classification effect of the strong classifier is further improved in the end [14]. The literature introduces methods to improve classification performance and proposes online learning algorithms. The insufficient Euclidean distance of the sample in a single specific subspace was checked. The literature introduces a pulse width modulation duty cycle control method that uses an integrator compensation method to obtain a higher PWM actuator accuracy at a lower frequency, which reduces the cost of PWM control technology [15, 16]. The motion control pulse closed-loop test experiment verifies the high performance and high precision of the design. The experimental verification of the motion control case shows the effectiveness of the design.

## 3. Theoretical Basis of Machine Learning and Distributed EM Algorithm

### 3.1. Machine Learning Algorithm

For example, the space label is set to *X*, which contains *m* styles *x*_*i*_ and the corresponding category label *ω*_*i*_. For the sake of simplicity, let it be a binary classification problem. There are a total of *K* weak classifications, which are *w*_*k*_, and their weights are weighted as *α*_*k*_ according to the classification effect of the weak classifications, which affects the weights of the weak classifications. The significant weight of the sample *D*_*k*__(*i*)_ satisfies formula (1). The initial weights are all the same.

(1) $$\begin{array}{c} \sum_{i=1}^{m}D_{k}\left(i\right)=1. \end{array}$$

In each training stage, the weak classifier *w*_*k*_ must be established to make it optimal for the samples with the weight distribution *D*_*k*(*i*)_. As shown in (2), in the process of learning weak classification, the goal is to reduce the loss function *ε*_*k*_.

(2) $$\begin{array}{c} \varepsilon_{k}=\sum_{i=1}^{m}P_{i□D_{k}\left(i\right)}\left[w_{k}\left(x_{i}\right)\neq \omega_{i}\right], \end{array}$$

where *P* [·] is the empirical probability observed in the training sample. This sample weak classification ratio will result in an increase in error, which is smaller than the error classification of the sample targeted by the weak classification *w*_*k*_. Therefore, the detector obtained through training is more effective than the random identification of the various components of the training sample set.

The expression *α*_*k*_ of the table weight is shown in

(3) $$\begin{array}{c} \alpha_{k}=\frac{1}{2}\text{ln}\left(\frac{1-\varepsilon_{k}}{\varepsilon_{k}}\right). \end{array}$$

The difference between online boosting and offline boosting is that the classifier must be trained online at each stage, and new samples must be used at each training stage. After updating the classifier, training samples will be deleted, offline boosting needs to prepare all training data in advance, and the classifier will not change after training. For the problem of tracking the target, due to the complexity of the target movement, if the classification cannot be changed and the target is constantly changing, the error may be more. Let the weak classifier be *w*_*k*_; the strong classifier is a linear combination of *K* weak classifiers; then, the confidence of the strong classifier can be expressed as

(4) $$\begin{array}{c} \text{conf}\left(x\right)=\sum_{k=1}^{K}\alpha_{k}w_{k}\left(x\right). \end{array}$$

In the online boosting target tracking algorithm, set *M* weak classifiers to form a weak classifier set, namely, *W*^weak ^={*w*_1_^weak ^,…, *w*_*M*_^weak ^}, set strong classifiers, select *K* weak classifiers from *M* weak classifiers, and select weak classifiers *W*^sel^ in

(5) $$\begin{array}{c} w^{\text{sel}}\left(x\right)=w_{m}^{\text{weak }}\left(x\right). \end{array}$$

Select the optimal feature vector corresponding to the weak classifier according to the following steps. As shown in formula (6), the weak classifier with the lowest misclassification rate is the selected weak classifier.

(6) $$\begin{array}{c} \text{arg}\underset{m}{\text{min}}\left(\varepsilon_{k,m}\right),\varepsilon_{k,m}=\frac{\lambda_{k,m}^{\text{wrong}}}{\lambda_{k,m}^{\text{corr}}+\lambda_{k,m}^{\text{wrong}}}. \end{array}$$

The final strong classifier is a linear combination of *K* weak classes, as shown in

(7) $$\begin{array}{c} S\left(x_{i}\right)=\text{sign}\left(\sum_{k=1}^{K}\alpha_{k}w_{k}\left(x_{i}\right)\right). \end{array}$$

The main advantage of the online learning tracking algorithm is that, when the algorithm is implemented, it only needs to identify the target and background information in a small area around the target to perform online update learning classification. However, this may cause problems in that after each update, different classifications may identify some tracking errors. The online semi-supervised boosting algorithm can effectively prevent the drift of the tracking process and can adapt to the continuous change of the target. The algorithm mainly combines prior knowledge and online learning courses to establish a process of updating the classifier in a semi-supervised manner.

The optimal feature vector determined by calculating the exponential loss function is shown in (8), which is the optimal weak classifier. Just look for the weak classifier that minimizes

(8) $$\begin{array}{c} L=\sum_{x\in X^{2}}e^{-js\left(x\right)}, \end{array}$$

where *L*_*X*_ is the sample set and *S* (*x*) is the strong classifier. The confidence measure that the sample is a positive sample is determined by

(9) $$\begin{array}{c} P\left(y=1|x\right)=\frac{e^{S\left(x\right)}}{e^{S\left(x\right)}+e^{-S\left(x\right)}}. \end{array}$$

In the semi-supervised offline learning boosting algorithm, the expression of the weak classifier and the weight of the algorithm are given in

(10) $$\begin{array}{c} w_{k}=\underset{w_{t}}{\text{argmin}}\left(\frac{1}{\left|X^{I}\right|}\sum_{x\in X^{L}}wl_{n}\left(x,y\right)-\underset{x\in X^{\prime }}{\sum }\left(p_{k}\left(x\right)-q_{k}\left(x\right)\right)\alpha_{k}w_{k}\left(x\right)\right), \end{array}$$

(11) $$\begin{array}{c} \alpha_{k}=\frac{1}{4}\text{ln}\left(\frac{1/X^{U}\left(\sum_{x\in X^{\prime }}p_{k}\left(x\right)+\sum_{x\in X^{\prime }}q_{k}\left(x\right)\right)+\left(1/X_{i}\left(x\right)=-1\right)\left(1/\left|X^{U}\right|\right)\left(\sum_{x\in X^{N}}q_{k}\left(x\right)+\sum_{x\in X^{\prime }}p_{k}\left(x\right)\right)+\left(1/x\in X^{L}\right)wl_{n}\left(x,y\right)}{|X_{i}\left(x\right)=y}\right). \end{array}$$

Among them, the probabilities of positive samples and negative samples in the unlabeled samples in (10) and (11) are the expressions (12) and (13) of *p*_*k*_ (*x*) and *q*_*k*_ (*x*), respectively.

(12) $$\begin{array}{c} p_{k}\left(x\right)=e^{-2S_{i-1}\left(x\right)}\frac{1}{X^{L}}\sum_{x,EX^{+}}Si\left(x,x_{i}\right)+\frac{1}{X^{U}}\underset{x,EX^{\prime }}{\sum }Si\left(x,x_{i}\right)e^{S_{t-1}\left(x\right)-S_{i-1}\left(x_{i}\right)}, \end{array}$$

(13) $$\begin{array}{c} q_{k}\left(x\right)=e^{2S_{i-1}\left(x\right)}\frac{1}{\left|X^{I}\right|}\sum_{x\in X^{-}}Si\left(x,x_{i}\right)+\frac{1}{\left|X^{U}\right|}\underset{x_{i}\in X^{\prime }}{\sum }Si\left(x,x_{i}\right)e^{S_{t-1}\left(x_{i}\right)-S_{i-1}\left(x\right)}. \end{array}$$

For positive samples, a positive sample classifier ∑_*x*∈*X*^+^_*S*^sim^(*x*, *x*_*i*_) ≈ *S*^+^(*x*) is obtained through learning and training to calculate the probability of *x* becoming a positive sample; the equivalent of ∑_*x*∈*X*^−^_*S*^sim^(*x*, *x*_*i*_) ≈ *S*^−^(*x*) is used to calculate the probability of *x* being a positive sample. In order to facilitate the distinction, a single strong classifier *S*^*p*^ is used here to identify positive samples and negative samples, *H*^+^ (*x*)∼*S*^*p*^ (*x*), that is, *H* (*x*)∼1 − *S*^*p*^ (*x*). According to formula (9) and the principle of boosting algorithm, formulas (11) and (12) can be simplified to

(14) $$\begin{array}{c} p_{k}\left(x\right)\approx \frac{e^{S_{k-1}\left(x\right)}e^{S^{p}\left(x\right)}}{e^{S^{p}\left(x\right)}+e^{-S^{p}\left(x\right)}}, \end{array}$$

(15) $$\begin{array}{c} {\tilde{q}}_{k}\left(x\right)\approx \frac{e^{S_{k-1}\left(x\right)}e^{-S^{p}\left(x\right)}}{e^{S^{p}\left(x\right)}+e^{-S^{p}\left(x\right)}}. \end{array}$$

The category *z*_*k*_ (*x*) of the unlabeled sample can be expressed as (15).

(16) $$\begin{array}{c} {\tilde{z}}_{k}\left(x\right)=p_{k}\left(x\right)-{\tilde{q}}_{k}\left(x\right)=\tanh\left(\left.H^{p}\left(x\right)\right)-\tanh\left(H_{k-1}\left(x\right)\right.\right). \end{array}$$

Combined with the online boosting algorithm, they proposed to decompose the target tracking problem into three parts: target detection, target recognition, and target tracking. These three parts are simplified and classified according to the integrity of the device itself. Target detection is responsible for finding the target of interest, target recognition distinguishes similar targets, and finally, target tracking is used to find the target.  Figure 1 shows the different parts of the algorithm.

### 3.2. Distributed EM Algorithm

The EM algorithm is an iterative method. For lost data, it is initially to solve the problem of estimating the parameters of the lost data. The main idea is first observe and analyze the data, and use the existing experience to estimate the value of the model parameters, then complete the estimation of the corresponding data value according to the estimated value of the parameter, and then by comparing the estimated missing value of the data with the previous value of the observed data. The value is added to estimate the value of the parameter, and the process is repeated until convergence; if the value does not change, the process will end. Therefore, the specific process of the algorithm is as follows:

Assuming that the set *X*={*x*_1_, *x*_2_, *x*_3_ … *x*_*m*_} of sample *X* follows the distribution of Gaussian mixture, the probability that the function *f*_*k*_(*x*) exists in the Gaussian mixture distribution is

(17) $$\begin{array}{c} f_{k}\left(x\right)=\sum_{j=1}^{k}w_{j}\Phi_{j}\left(x_{i};\theta_{j}\right). \end{array}$$

Among them, the Gaussian element with probability Φ_*j*_(*x*_*i*_; *θ*_*j*_) is expressed as

(18) $$\begin{array}{c} \Phi_{j}\left(x_{i};\mu_{j},\Sigma_{j}\right)=\frac{\exp\left\{-1/2{\left(x_{i}-\mu_{j}\right)}^{T}\sum_{k}^{-1}\left(x_{i}-\mu_{j}\right)\right\}}{{\left(2\pi \right)}^{p/2}{\left|\Sigma_{k}\right|}^{1/2}}. \end{array}$$

Given the initial value *μ*_0_, Σ_0_, *w*_0_, repeat Steps 1 and 2 until they converge.

**Step 1 .**

Calculate the probability of the recessive variable according to the initial value of the parameter *θ* as the current estimated value of the recessive variable:

(19) $$\begin{array}{c} Q_{i}\left(z^{\left(i\right)}\right)≔f\left(z^{\left(i\right)}Lx^{\left(i\right)};\theta \right). \end{array}$$

**Step 2 .**

Obtain new parameter values by calculating the maximum value of the estimation function:

(20) $$\begin{array}{c} \theta ≔\text{arg}\underset{\theta }{\text{max}}\sum \sum_{i,z^{\left(i\right)}}Q_{i}\left(z^{\left(i\right)}\right)\log\frac{f\left(x^{\left(i\right)},z^{\left(i\right)};\theta \right)}{Q_{i}\left(z^{\left(i\right)}\right)}. \end{array}$$

Finally obtain

(21) $$\begin{array}{c} w_{k}^{t+1}=\frac{\sum_{i=1}^{n}f\left(k|x_{i},\theta^{t+1}\right)}{n},\\ \mu_{k}^{t+1}=\frac{\sum_{i=1}^{n}f\left(k|x_{i},\theta^{t+1}\right)x_{i}}{\sum_{i=1}^{n}f\left(k|x_{i},\theta^{t+1}\right)},\\ \sum_{k}^{t+1}=\frac{\sum_{i=1}^{n}f\left(k|x_{i},\theta^{t+1}\right)\left(x_{i}-\mu_{k}^{t+1}\right){\left(x_{i}-\mu_{k}^{t+1}\right)}^{T}}{\sum_{i=1}^{n}f\left(k|x_{i},\theta^{t+1}\right)}. \end{array}$$

Finally, by calculating the parameter values, each sample can be found and the final result of the grouping can be obtained.

When using machine learning algorithms, we must first consider the accuracy and efficiency of the algorithm. The traditional EM algorithm has defects in these two aspects. This makes the algorithm more sensitive to the initial values of the parameters, which leads to the convergence result easily falling into the local optimum of the likelihood function. In addition, the traditional EM algorithm uses an iterative calculation method, which leads to the need to load data multiple times. Therefore, the specific direction for optimizing the EM algorithm at this stage is how to effectively solve these two problems: (1) the number of initial components that need to be manually set in the model and (2) as the data size increases, the convergence speed decreases rapidly.

Based on the calculated density of the original probability *f*_*k*_(*x*) in the Gaussian distribution mixed by the EM algorithm, the new component *δ* (*x*; *θ* is added to the existing density function *f*_*k*_(*x*) of the *k*-component mixture, and the density function of the Gaussian mixture model is as follows:

(22) $$\begin{array}{c} f_{k+1}\left(x\right)=\left(1-\alpha \right)f_{k}\left(x\right)+\alpha \delta \left(x;\theta \right). \end{array}$$

Then, the newly generated log-likelihood function is

(23) $$\begin{array}{c} L_{k+1}=\sum_{i=1}^{n}\text{log}\left[\left(1-\alpha \right)f_{k}\left(x\right)+\alpha \delta \left(x;\theta \right)\right]. \end{array}$$

Extend Taylor's second-order formula *L*_*k*+1_ to *α*_0_ and maximize the quadratic function of *α* to obtain an approximate value of the probability of action:

(24) $$\begin{array}{c} L_{k+1}^{\wedge }=L_{k+1}\left(\alpha_{0}\right)-\frac{{\left[L_{k+1}^{\prime }\left(\alpha_{0}\right)\right]}^{2}}{2L0_{k+1}^{\prime \prime }\left(\alpha_{0}\right)}. \end{array}$$

Here, *L*_*k*+1_′ and *L*_*k*+1_^″^ are the first and second derivatives of *α*.

(25) $$\begin{array}{c} \chi \left(x;\theta \right)=\frac{f_{k}\left(x\right)-\delta \left(x;\theta \right)}{f_{k}\left(x\right)+\delta \left(x;\theta \right)}. \end{array}$$

Then, the log-likelihood local optimal can be written as

(26) $$\begin{array}{c} L_{k+1}^{\wedge }=\sum_{i=1}^{n}\text{log}\frac{f_{k}\left(x_{i}\right)+\delta \left(x_{i};\theta \right)}{2}+\frac{1}{2}\frac{{\left[\sum_{i=1}^{n}\chi \left(x_{i};\theta \right)\right]}^{2}}{\sum_{i=1}^{n}\chi^{2}\left(x_{i};\theta \right)}. \end{array}$$

From this, the formula for *α* can be obtained:

(27) $$\begin{array}{c} \hat{\alpha }=\frac{1}{2}-\frac{1}{2}\frac{\sum_{i=1}^{n}\chi \left(x;\theta \right)}{\sum_{i=1}^{n}\chi^{2}\left(x;\theta \right)}. \end{array}$$

In this way, the optimal solution {*α*_*k*+1_, *μ*_*k*+1_, Σ_*k*+1_} of the new model parameters can be obtained. The value of the logarithmic function of the probability in the Gaussian mixture model is *L*_*k*+1_.

### 3.3. Algorithm Simulation

In order to prove the stability and effectiveness of the tracking algorithm in this chapter, this chapter conducts a series of experiments to verify the algorithm. The experiment is divided into 3 groups. The targets of the three videos are running car, David in door, and occluded face. The comparison experiment uses the original MIL and TLD algorithms. The tracking error in the algorithm experiment uses the calculated target position and the Euclidean distance from the actual target position.

**Experiment 1 .**

Part of the experimental results of running car video sequence. There are 5 cars in the video, and some are very similar. During the movement, the car often makes actions that interfere with the tracking, and the road and the camera itself also interfere with the tracking of the target. In this experimental tracking process, the consistency of the target is very high in the first 200 frames and about 400 frames. The tracking frame of the TLD algorithm is between the blocked target and the actual target beating back and forth. In the next sequence, the interference of the same object will become smaller. At this time, TLD tracking is relatively stable. When the target is disturbed, the algorithm does not seem to jump and can maintain stability, and the original MIL algorithm shows two shortcomings in the tracking process. First of all, the tracking speed is very slow and cannot fully meet the requirements in real time. On the other hand, as the time changes in the tracking process, the drift of the frame is also increasing, which eventually leads to failure. Experiments show that the processing speed of the algorithm is not only higher than the original algorithm, but also can track the target stably under certain interference conditions.  Figure 2 shows a graph comparing the tracking errors of these three algorithms. It can be seen from the figure that when the target reaches about 250 frames, there is a little drift guide for the first time, and the tracking has been relatively stable since then.

**Experiment 2 .**

Compare the processing speed of the original algorithm with the algorithm. From the algorithm error comparison chart in Figure 3, it can be seen that the algorithm is always the tracking algorithm with the smallest error in the first 390 frames. Finally, the cumulative error is too large, so it makes the drift trace larger.

**Experiment 3 .**

Occluded face tracking experiment, a total of 819 frames. The tracking target first does not move in the field of view and then covers his left face with a book. Then, he lowered his head and covered the right half of his face with a book. Then, he sat upright, put on his hat, and covered his hair and forehead. Then, he covered the lower half of his face with a book, showing only his eyes. The final goal was to drop the book. In the 250th frame of the tracking process, the target covers the left face with the book, and the original MIL algorithm cannot identify the value between the positive samples. Therefore, when the book covers the face, it will always be used as the background, so the tracking starts to drift. If you remove the book, the tracking frame will still not return to the target position, but always treat the calculated position as the actual target position. Similarly, when the book covers the right side, the trace of the frame starts to move to the left and will not return to the correct trace. At frame 700, the target first puts on a hat and then covers his face. In this group of experiments, it can be concluded that compared with other algorithms, the effectiveness of this algorithm has been greatly improved. From the comparison error tracking diagram of the three algorithms in Figure 4, it can be seen that the algorithm does not produce too much error for all 819 consecutive data frames of video tracking and can be tracked stably.

#### 3.3.1. Experimental Environment

The entire experiment is performed under the Hadoop platform, each host system uses Ubuntu 14.04, and the Java environment is OpenJDK 7.  Table 1 shows the configuration of the Hadoop cluster nodes.

#### 3.3.2. Experimental Results and Analysis

The experimental data come from the iris plant data set placed in the standard UCI test database. The data have 4 attributes: characteristic information about sepal length, sepal width, petal length, and petal width. The four attributes are in centimeters. Each set of data has examples.

*(1) Run Time Comparison*. In the process of processing the data set, this algorithm is time-consuming to compare with the other two algorithms. The result obtained is shown in Figure 5.

By grouping the data, it can be seen from the figure that the grouping result is correct. And compared with the other two algorithms, the algorithm consumes significantly less time when processing data sets and has good scalability. Scalability of the algorithm: By changing the number of nodes, set the number of nodes to 2, 4, 6, and 8, respectively, and observe the changes in the processing time of the iris plant data placed under the algorithm. The experimental results are shown in Figure 6.

It can be seen from the figure that the number of nodes is inversely proportional to the running time of the algorithm, so the running speed of the algorithm can be improved by increasing the number of nodes for calculation. At the same time, if the data set is small due to the increase in the number of nodes, the running time of the algorithm will be very short. This is because under a small data scale, the calculation time of the iterative algorithm is very small, and most of the time is spent on node-to-node communication. Finally, these two experiments confirmed that the algorithm improves the processing efficiency of multiple data sets, while ensuring the accurate output of multiple components in the model. The processing speed of the algorithm can be further improved by increasing the number of nodes, and it has good system scalability.

## 4. Design and Practical Application of Movement Visualization System

### 4.1. Hardware Design of Motion Visualization System

It draws a block diagram of the working principle of PLC motion control. The high-speed computer writes the motion control program and downloads it to the PLC. The servo motor drives the parts to move. It always has an internal code input, and the servo ensures that the control pulse command issued by the PLC is executed according to the feedback of the encoder.

Motion control consists of several key points, including the origin and the limit position of forward and reverse rotation. From a safety point of view, two extreme positions are set in the forward and reverse rotation, and there are two extreme positions. If the mechanical movement reaches the limit of the forward rotation program, it will move to the mechanical limit before reaching the limit. Or, if the forward movement exceeds the reverse limit of the program and reaches the mechanical limit, it must be decelerated; otherwise, electrical damage may occur due to over speed exceeding the mechanical limit. Before reaching the forward rotation limit 2 or the reverse rotation limit 2, you must stop immediately; otherwise, the mechanical position will be damaged. The forward rotation or reverse mechanical limit of the mechanical limit is the farthest point that can reach the moving mechanical mechanism; otherwise, the mechanical or electrical equipment will be damaged.

In order to complete the practical application of motion control instructions, the designed instruction set requires specific scientific. First, the instruction set must be complete, allowing users to work together freely to obtain the control requirements of different applications; second, the single function of the instruction should not be too simple, in this case. If it is too simple, you need to complete multiple instruction combinations to complete, and the amount of programming is large. The overly complex instructions are highly professional. It is not easy to combine to meet the needs of different applications.

The coding system of the PLC command system is very important. The instructions in this article use general standard programming language technology to achieve basic standard instructions, and the programming style also meets the requirements. Among them, because the IEC61131-3 PLC standard program is widely used worldwide, many engineers are familiar with the use of PLC instructions. Most engineers are easy to accept programmable controllers containing typical motion control instructions and are compatible with PLC motion control technology solutions. They are extremely versatile and can be developed for applications. The software is highly adaptable, easy to install, and easy to develop. The PLC standard is an international standard. It will continue to research and expand on the basis of the meter standard, and will continue to promote technological development through the industry, thereby gaining market recognition and acceptance.

### 4.2. Motion Command Processing

The solution is based on the translated PLC instructions, and the motion control instructions are implemented separately in internal processing. The PLC designed in this article uses a 32-bit ARM chip architecture. In the architecture scheme, the instructions for encoding and scanning instructions fully consider the characteristics of the 32-bit chip. Designing a 32-bit encoding format can further improve the speed of PLC instructions. The execution of the instruction is divided into three stages: take over the instruction, execute the instruction, write back, etc. The command code indicates the function code in the command. According to different command codes, the command may have multiple variable parameters. The instruction format is shown in Table 2, which is used to display the execution behavior of the instruction.

This parameter is composed of several bytes, and its format is shown in Table 3. Smaller digital offset indicates that there is a small offset in some parameters, and the storage area corresponds to each storage area number code used by the PLC.

Immediate variable, that is, a 4-byte value, format is shown in Table 4.

For example, if the button is pressed, the simple initial return execution plan, %IX0.0, obtains the input signal, and the program in the instruction list used to execute the initial return function has two sentences. The intermediate code of the translation result is shown in Table 5.

Select the IL instruction list language selected by the IEC61131-3 standard as the intermediate language, and change the ladder diagram to the instruction list language. The IL instruction list plays an important role as an assembly bridge for the entire language of the IEC61131-3 standard. Then, the ladder diagram is converted into the language of the instruction list. The key problem to be solved in the conversion process from the ladder diagram to the instruction list is the data storage structure of each node in the ladder network and the identification of the interconnection between the nodes. The problem of the maze is a classic problem in the field of graphics and graph theory. In this chapter, the idea of solving the maze problem is applied to transform the ladder diagram into a statement list. After the binary tree of the series relationship is established, the network scale map is scanned through the expanded maze algorithm to determine the left and right connection relationship of the original node, and a two-way binding list of the original node is created. The double-linked nodes in the list are identified by identifying serial and parallel connections to identify each node in the list that is linked to the binary tree; finally, the binary tree is traversed and the instruction list statement is output. The algorithm avoids special situations such as virtual nodes, and the algorithm processing greatly reduces the complexity of the algorithm and ensures the efficiency and accuracy of algorithm modification.

A ladder program is composed of several ladder networks. Each scale network contains multiple graphical node elements. Each graphic element node occupies an area the size of a rectangle. Among them are graphic symbols that show the differences between nodes. No area on the node is empty. The ladder node diagram described in this article contains symbols and primitive node types, as shown in Table 6.

### 4.3. The Value of Visual Teaching

On the basis of the comprehensive development of students' comprehensive abilities and the requirements of meeting their lifelong development needs, our country has implemented a new curriculum reform. In the new curriculum reform, my country strongly supports quality education. Physical education is an important course to improve the health of students, and it is widely concerned by the state. With the rapid development of science and technology and the enhancement of people's ability to apply science and technology, in order to better implement the new curriculum reform supported by the state, our country has introduced modern information teaching technology. It visualizes knowledge and provides more possibilities for teaching. Therefore, the application of modern teaching information technology in physical education courses is gradually being promoted and used. Movement visualization exercise teaching is an important way to use modern technology to teach information in contemporary physical education courses. It has multiple values in the physical education curriculum.

## 5. Conclusion

This article studies the related theories of machine learning and target tracking technology, which is an important field of computer vision research and is widely used in a variety of situations (such as military and civilian fields). Especially in military analysis, on-site monitoring, firepower strikes, etc., it all plays an important role. With the expansion of the tracking range, the difficulties encountered in practical application of this technology have gradually increased. In recent research directions, machine learning-based target tracking technology has become a tracking strategy in the future. This allows the computer to adjust the position of the tracker at any time according to changes in the target. Maintain stable target tracking.

With the development of big data technology research, how to use big data technology to optimize traditional clustering analysis algorithms and improve the ability to process multiple data sets has become a topic. This technology can help people easily extract important information from large amounts of data so as to meet the needs of contemporary people to obtain and exchange information, which has also become the focus of academic and industrial research. In the context of multi-data search and machine learning algorithms, this article starts with an introductory problem of mainstream big data technology MapReduce rendering framework and EM value. Research on the management of a large amount of data, on this basis, is based on the relevant data; this paper proposes a greedy EM algorithm. The algorithm can ensure that the number of initial components of the model does not have to be determined in advance, and the number of components of the model can be retrieved correctly, thereby further improving the processing and convergence speed of multiple data sets.

## Figures and Tables

**Figure 1:** Beyond semi-supervised tracking algorithm composition.

**Figure 2:** Running car video sequence tracking error comparison curve.

**Figure 3:** David in door video sequence tracking error comparison curve.

**Figure 4:** Occluded face video sequence tracking error comparison curve.

**Figure 5:** Algorithm running time comparison chart.

**Figure 6:** Algorithm running time under different nodes.

**Table 1:** Hadoop cluster node configuration.

Numbering	Node name	CPU name	IP address
01	Master	Hadoop	192.168.168.32
02	Slaver l	Hadoop 1	192.168.168.33
03	Slaver 2	Hadoop 2	192.168.168.34
04	Slaver 3	Hadoop 3	192.168.168.35
…	…	…	…
08	Slaver 7	Hadoop 7	192.168.168.39

**Table 2:** PLC instruction format.

Differential	Immediate	Keep
2 (bit)	1 (bit)	5 (bit)

**Table 3:** Format of double-byte parameter variable.

4 bit	4 bits	1 byte	1 byte
Bit shift	Storage area	Low word high byte of storage area	Low word low byte of storage area

**Table 4:** Format of immediate parameter variable.

2 bytes	2 bytes
High word	Low word

**Table 5:** Example of PLC motion control instruction code format.

Instruction list statement	Significance	Command code	Instruction format	Parameter format	Parameter
LD%IX0. 0	Load input contact% 1 × 0.0	0100	00	00	030000
DSZR 0	Perform home return	0020	00	00	000000

**Table 6:** The meaning of the primitive node type.

Primitive node symbol	Node type	The meaning of the node	The role of nodes in the ladder diagram
(blank)	Empty node	No nodes here	Blank means there are no primitives here
—	Connection line	Horizontal connection line	Connect two primitive nodes horizontally
丨	Connection line	Vertical connection line	Vertically connect two primitive nodes
卄	Real node	Contacts	Input component
<)	Real node	Coil	Output-type components

## Data Availability

The data used to support the findings of this study are available from the corresponding author upon request.
